# Comparison of the Interrupted and Continuous Suture Techniques for the Closure of Oral and Nasal Mucosal Layers in Cleft Palate Surgery

**DOI:** 10.7759/cureus.20779

**Published:** 2021-12-28

**Authors:** Owais Ahmed, Yusra Afzal, Mirza Shehab A Beg, Aimen S Siddiqui, Farkhandah M Iqbal

**Affiliations:** 1 Plastic and Reconstructive Surgery, Liaquat National Hospital and Medical College, Karachi, PAK; 2 Plastic Surgery, Liaquat National Hospital, Karachi, PAK

**Keywords:** number of suture packs, operative time, palatal fistula, nasal and oral layer, palatal repair, interrupted vs continuous

## Abstract

Background

Cleft lip and palate are common congenital craniofacial anomalies, treated conventionally by surgery at the ages of six to 18 months. Mostly, the interrupted suture technique is used to close the nasal and oral layers of the palate. In some studies, the interrupted suture technique was compared with continuous suture techniques for the closure of oral and nasal layers and found that there was less utilization of time and suture materials in the continuous technique. This study was designed to see the outcomes of interrupted versus continuous suture techniques.

Materials & methods

A total of 36 patients were included in the study and were divided into two groups according to the type of suturing technique. The time utilized for the repair of the oral and nasal layers of the cleft palate, the number of suture packs utilized, and the incidence of fistula formation were noted and compared between the two groups. Out of 36 patients, 17 were included in group A (operated by interrupted techniques), and 19 were included in group B (operated by the continuous technique).

Results

The mean time taken to close nasal layer in Group A was 18.12 ± 1.16 minutes and in Group B was 8.37 ± 0.89 minutes (p-value < 0.001), whereas for oral layer closure, it was 14.00 ± 1.17 minutes in group A and 6.00 ± 0.57 minutes in group B (p-value < 0.001). The average usage was 2.26 ± 0.45 suture packs for repair with the continuous technique and 4.00 ± 0.35 suture packs when repaired via interrupted stitches. There was no difference noted in postoperative outcomes in both groups in terms of postoperative fistula and wound dehiscence.

Conclusion

A continuous suture technique for closing the oral and nasal layers in patients with cleft palate is recommended, as it is more beneficial in terms of time, cost-effectiveness, and utilization of suture material.

## Introduction

Cleft lip and palate are common congenital craniofacial anomalies treated by plastic surgeons [1]. The incidence of cleft lip and/or cleft palate is 1.91 per 1000 live births (one in 523 live births) in Asians [2]. A cleft palate would result in feeding difficulties, speech problems, hearing difficulties, and dental abnormalities if left untreated.

In cleft palate repair, the primary objective is to regain the anatomic oro-nasal continence and to establish the normal velopharyngeal mechanism. There are multiple well-established techniques being used for cleft palate repair; they differ in terms of dissection method, incision site, and flap elevation. The palate is traditionally repaired by closing oral and nasal layers separately with interrupted sutures between the ages of six and 18 months [3]. The techniques of cleft palate repair are continuously evolving with some surgeons focusing on the repair of oral and nasal layers via continuous or running stitches [4]. The oro-nasal fistula is the main complication of palatoplasty. The incidence varies from less than 2% to over 40% in different published studies [5].

A study described the advantage of the continuous suture over the interrupted suture in terms of efficiency and cost-effectiveness in the face and neck regions [5]. In some other studies, it was concluded that the continuous suture requires less time and suture materials to close a similar length of the palate when compared with the interrupted suture [5-6]. Generally, continuous stitches are known to compromise vascularity and increase the chances of wound dehiscence [1]. This disadvantage has less importance for the region of the head and neck, as the blood supply is robust as compared to other regions of the body [2]. The usage of continuous sutures for the closure of the nasal and oral layers of cleft palate is reported in a few studies only based on the individual practice of surgeons [2].

This comparative study was designed at our center to evaluate the effectiveness of continuous sutures for closing the nasal and oral mucosa in cleft palate repair and compare it with the interrupted suturing techniques in terms of total operative time, number of suture packs utilized, and outcomes of the procedure, including postoperative wound dehiscence and fistula formation.

## Materials and methods

This study was conducted at the department of plastic and reconstructive surgery, Liaquat National Hospital, Karachi, between July 2020 and April 2021. Prior approval was taken from the institutional review committee with approval number App # 0573-2021-LNH-ERC; informed assent for inclusion in the study was obtained from patients' parents and they were briefed about the nature and purpose of the study.

All male/female patients operated for unilateral or bilateral cleft palate, from six to 18 months of age were included in the study. Patients above 18 months of age, previously operated for cleft palate, with palatal fistula, and with syndromes or comorbidities were excluded from the study. Demographic data were documented at the time of initial presentation and patients were assigned to either group A (interrupted suture) or group B (continuous suture) by the non-probability sampling technique.

All the patients were operated on by consultant plastic surgeons with more than 20 years of experience in cleft surgery. The standard Bardach technique used for palate repair [7], in which mucoperiosteal flaps are raised bilaterally based on the greater palatine vessel, nasal layers released, muscles separated from the bone, the defect of the soft palate was closed in three layers with intravelar veloplasty and of the hard palate in two layers. For closing the nasal and mucosal layers, either of the two suture techniques, continuous or interrupted, was used. An illustration of nasal and oral layer closure is shown in Figures 1-2 (continuous technique) and Figure 3 (interrupted technique).

**Figure 1:** Cleft palate repair - continuous suture technique 1-A: Cleft palate (preoperative picture) 1-B: The nasal layer of the cleft palate repaired via continuous suture technique (patient 1)

**Figure 2:** Cleft palate repair - continuous suture technique 2-A: The oral layer of the cleft palate - repaired via continuous suture technique (patient 1) 2-B: The oral layer of the cleft palate - repaired via continuous suture technique (patient 2) - closed view

**Figure 3:** Cleft palate repair: interrupted suture technique 3-A: Cleft palate 3-B: The cleft palate repaired via the interrupted suture technique (patient 3)

Similar suture material and length were used in all the patients. Recordings like operative time (the time taken to close the oral and nasal layers of the palate) in minutes were documented using a stopwatch. The time utilized for the dissection of the palate was not included in the operative time, as it may vary due to different levels of difficulty, depending upon the varied anatomy and bleeding. The number of suture packs used to close the nasal and oral layers was noted at the end of the procedure. Postoperatively, patients were examined in the outpatient department to look for fistula formation and wound dehiscence. The minimum follow-up time was three months for all the patients. All the data were documented in a predesigned proforma. Photographic records of every patient were maintained after taking assent from the patient's parents.

Statistical analysis

Data were entered and analyzed by using SPSS version 25 (IBM Corp., Armonk, NY). Mean and standard deviation was computed for the quantitative variables. Frequency and percentage were calculated for qualitative variables. Association of the fistula with treatment groups was done using the chi-square test and considering p-value ≤ 0.05 as significant. Differences in age, nasal layer closure time, and oral layer closure between the treatment groups were compared using an independent t-test (p-value ≤ 0.05 taken as significant).

## Results

The total number of cleft palate patients enrolled in this study was 36. Group A consisted of patients whose oral and nasal layers were repaired with interrupted suturing while Group B with continuous suturing. Group A (interrupted) had 17 patients (47.2%) while Group B (continuous) had 19 patients (52%) (Figure 4).

**Figure 4:** Total number of patients in each group

The mean age of the study population in Group A was 10.88 ± 1.93 months while in Group B, it was 10.63 ± 1.57 months. The male-to-female ratio in Group A was 1:1.12 while in Group B, it was 1.37:1. Descriptive statistics of the study population are mentioned in Table 1.

**Table 1:** Descriptive statistics of the study population Gender-wise distribution of subjects and frequency of the type of clefts (uni/bilateral)

		Group A (Interrupted) N (%)	Group B (Continuous) N (%)
GENDER	Male	8 (47.1%)	11 (57.9%)
	Female	9 (52.9%)	8 (42.1%)
CLEFT TYPE	Unilateral	9 (52.9%)	10 (52.6%)
	Bilateral	8 (47.1%)	9 (47.4%)

The incidence of the palatal fistula was found to be more or less similar in both groups. By applying the chi-square test, no statistical significance was noted (p-value = 0.935) (Table 2).

**Table 2:** Comparison of incidence of palatal fistulas between treatment groups

	Group A (Interrupted) N (%)	Group B (Continuous) N (%)	p-Value* Chi-Square Test
YES	1 (5.9%)	1 (5.3%)	0.935
NO	16 (94.1%)	18 (94.7%)	
*p-value < 0.05			

The mean time taken for nasal and oral layer closure in Group B (continuous suturing techniques) was much less than that of Group A (interrupted suturing technique) and was found to be statistically significant when the chi-square test was applied, that is, for the oral layer (p <0.001) and for the mucosal layer (p<0.001) (Table 3).

**Table 3:** Comparison of mean time (minutes) taken to close the oral and nasal layers of the cleft palate

	Group A (Interrupted) Mean ± SD (minutes)	Group B (Continuous) Mean ± SD (minutes)
Time of nasal layer closure	18.12 ± 1.16	8.37 ± 0.89
Time of oral layer closure	14.00 ± 1.17	6.00 ± 0.57

The average number of suture packs utilized for the repair of oral and nasal layers of the cleft palate with the continuous technique was 2.26 ± 0.45 while 4.00 ± 0.35 suture packs were utilized when repaired via interrupted stitches; they were compared by using the chi-square test and found to be statistically significant (p-value <0.001) (Table 4).

**Table 4:** Average number of suture packs utilized for each group

	Group A (Interrupted) Mean ± SD	Group B (Continuous) Mean ± SD
Number of sutures packs utilized	4.00 ± 0.35	2.26 ± 0.45

## Discussion

The occurrence of cleft palate shows interesting racial predilections, seen more commonly in Asians [8], and therefore its management in terms of early diagnosis and appropriate surgical intervention adds substantially to the health care burden in Pakistan [3]. A multidisciplinary approach is required for caring for the child with a cleft palate that starts with prenatal diagnosis (where available), evaluation for other possible congenital anomalies, decisions about the timing of repair and choice of techniques [9], and continuing into adulthood for the secondary procedure when needed [3]. Pre and postoperative management of these cleft patients must also include a multidisciplinary team consisting of an otorhinolaryngologist, an orthodontist, a speech therapist, and a pediatrician to manage overall health and nutrition [9]. Although the prime answer to the care of the cleft patient is surgery some techniques may improve the surgical outcomes done in infancy like presurgical nasal-alveolar molding (NAM) [10].

Several surgical techniques have been described in the literature to address cleft patients. A survey from cleft surgeons affirms that the Bardach two-flap palatoplasty with intravelar veloplasty and the Furlow double-opposing z-plasty were the two most commonly used techniques for palate repair, accounting for 87 percent of all cases [11]. Traditionally, the palate is repaired with interrupted sutures. 

This study was designed to compare the effects of continuous versus interrupted sutures in terms of time required for suturing, length of suture threads used, and rates of postoperative complications like wound dehiscence and oro-nasal fistula.

In the past years, there is no improvement in the care of orofacial clefts. Therefore, strategic cooperation between countries to compare and contrast diverse treatment conventions and surgical techniques can deliver more reliable, consistent, and predictable results [12]. Despite many advancements in the medical field, the choice for suturing via the continuous or interrupted technique remains controversial. There is a continuous discussion as to which suturing procedure best accomplishes definitive wound closure in a more precise time with minimum complications [13]. According to multiple studies, there is a considerable reduction in surgical time when continuous sutures were applied as opposed to interrupted sutures [5]. This is especially true for a single surgeon with no suturing assistance because of the tight space in the oral cavity. This technique is quite simple to perform and does not require individual knots for each suture, which makes the whole process of suturing the oral and nasal mucosal layers a lot faster. In a recent study of 152 cleft palate patients, it is reported that the mean time taken for nasal layer closure by continuous sutures was 7.08 ± 1.19 minutes, whereas, for interrupted sutures, it was 11.50 ± 1.16 minutes [3]. Similarly, for oral layer closure, it took a mean duration of 17.90 ± 2.09 minutes with the continuous suturing technique and 19.23 ± 1.48 minutes with the interrupted suturing technique [3]. The results of our study correlate with the results of the above-mentioned study, that is, the mean time taken for nasal layer closure by continuous sutures was 8.37 ± 0.89 minutes while it was 18.12 ± 1.16 minutes for interrupted sutures, and for oral layer closure, it took a mean duration of 6.00 ± 0.57 minutes with the continuous suturing technique and 14.00 ± 1.17 minutes with the interrupted suturing technique. This brief analysis demonstrates a clear advantage of using continuous sutures over interrupted sutures, concerning time consumed during the procedure. This, in turn, saves total anesthetic and surgical time and hence contributes heavily toward saving total operation theatre costs. This is especially beneficial for a country with low revenue like Pakistan.

Repair via the continuous technique uses up less amount of suture material in comparison to the interrupted suture technique, as only two knots are tied (one packet compared to two or three packets, respectively, in some different types of wounds) [6]. The study by GQ Fayyaz et al. reported the average usage of 2.12 ± 0.33 suture packets for the continuous suture group and 4.59 ± 0.49 for the interrupted suture group [3] while in our study, the average usage was 2.26 ± 0.45 suture packs for repair with the continuous technique and 4.00 ± 0.35 suture packs when repaired via interrupted stitches. This shows that the interrupted suture technique utilizes roughly double the amount of suture material used for the continuous suture technique. The cost savings obtained by the continuous suturing pattern for individual palatoplasty procedures may not quantify to a considerable amount but when extrapolated to a hospital or the national level, they constitute an impressive sum of the health care budget. Keeping in mind the economic burden associated with the high incidence of cleft palate cases every year in our country, a preference for the continuous suturing technique can enable hospitals to narrow down surgical costs and manage funds more efficiently.

One criticism of the continuous suturing pattern is that if the suture breaks at any point, the integrity of the whole palate will be compromised, as only a single suturing thread is used. This is not seen in the interrupted technique as individual sutures along the palate are not connected. Instead of using a single thread to pull the palate edges closed, interrupted sutures comprise numerous stitches placed close together, which disseminate tension more equitably over the length of the palate and make the difference to keep the cleft palate from becoming separated in case of rupture of even a single suture [3]. In our study, we applied one interrupted sutures at each end of the repair for additional support to the continuous sutures to minimize the risk of palate dehiscence, however, we didn't find a single case of dehiscence in patients repaired via the continuous suture technique.

Cleft palate repair surgery may be followed by challenges like bleeding, respiratory distress, infections, and dehiscence but the most commonly reported post-surgical complication is the formation of oronasal fistula [14]. The incidence of fistula formation after cleft palate repair varies between 5% and 34%. Technical failure resulting from poor surgical technique, tense closure, infections, foreign body irritation, absent multilayer repair, and poor healing contributes to oro-nasal fistula formation [14-15]. According to a study published by GQ Fayyaz, the occurrence of the fistula was almost equal in both the continuous and interrupted suture groups [3]. However, in our study, its frequency was also similar when the cleft palate was repaired via interrupted (5.9%) or continuous (5.3%) sutures. But further studies are needed to directly correlate the association between the two factors.

There were a few limitations of this study. The sample size was small and the age group was very narrow. It is highly recommended that further studies be conducted on other varieties of cleft palate, different age groups, and with a large sample size to increase the trust in continuous suturing in palate surgery.

## Conclusions

Continuous sutures for the repair of cleft palates save operative time and effort of the surgeon while operating in deep tight spaces, reduce the amount of suture material as compared to interrupted sutures, and an increased risk of postoperative complications in terms of wound dehiscence or fistula formation is absent. We suggest that for cleft palate repair, continuous suturing can be used as a standard technique.
